# A Computational Intelligence Model for Legal Prediction and Decision Support

**DOI:** 10.1155/2022/5795189

**Published:** 2022-06-24

**Authors:** Xuerui Shang

**Affiliations:** School of Law, Shanghai University of Finance and Economics, Shanghai, 200433, China

## Abstract

Legal judgment prediction (LJP) and decision support aim to enable machines to predict the verdict of legal cases after reading the description of facts, which is an application of artificial intelligence in the legal field. This paper proposes a legal judgment prediction model based on process supervision for the sequential dependence of each subtask in the legal judgment prediction task. Experimental results verify the effectiveness of the model framework and process monitoring mechanism adopted in this model. First, the convolutional neural network (CNN) algorithm was used to extract text features, and the principal component analysis (PCA) algorithm was used to reduce the dimension of data features. Next, the prediction model based on process supervision is proposed for the first time. When modeling the dependency relationship between sequential sub-data sets, process supervision is introduced to ensure the accuracy of the obtained dependency information, and genetic algorithm (GA) is introduced to optimize the parameters so as to improve the final prediction performance. Compared to our benchmark method, our algorithm achieved the best results on four different legal open data sets (CAIL2018_Small, CAIL2018_Large, CAIL2019_Small, and CAIL2019_Large). The realization of automatic prediction of legal judgment can not only assist judges, lawyers, and other professionals to make more efficient legal judgment but also provide legal aid for people who lack legal expertise.

## 1. Introduction

In traditional judicial cases, the results can be obtained only after the analysis and interpretation of relevant people, and the complexity and professionalism of legal documents are insurmountable barriers for ordinary people. In early studies, relevant people build expert systems in the judicial field to solve the problems encountered by people, but in the construction process of expert systems, legal people often need to provide a lot of rules and definitions, and the later maintenance of the system will consume a lot of time and energy. With the maturity of deep learning technology, a large number of excellent deep neural network models have been proposed, which lays a solid foundation for intelligent judicial research. Article prediction is an important subtask in intelligent justice. The article prediction task can assist judges to deal with cases; predict the law involved in the trial process, provide the basis for the judicial decision of charges, prison terms, fines, and so on; and greatly improve the efficiency of judges to deal with cases. Legal judgment prediction (LJP) tends to enable machines to forecast the verdict of legal cases after reading the description of facts, which is an application of AI in the legal field. The realization of automatic prediction of legal judgment can not only assist judges, lawyers, and other professionals to make more efficient legal judgment but also provide legal aid for people who lack legal expertise. Recently, with the development of machine learning and natural language processing (NLP) technology, the research on the prediction of legal decisions has attracted more and more scholars' attention.

LJP research began decades ago [1–5]. At present, the legal judgment task is regarded as text classification task. Researchers have carried out researches on this task and proposed many landmark methods [6–13], mainly including the traditional machine learning method and deep neural network-based legal judgment prediction method. Most of the legal judgment methods [9, 10] based on traditional machine learning methods mark features manually based on specific case types, which are difficult to be applied to other types of cases and have poor adaptability to scenarios. The legal judgment prediction method [11, 12] based on the deep neural network no longer relies on the manual carefully designed template but captures the context information through the convolutional neural network or cyclic neural network and makes feature representation according to the description of the case facts so as to achieve judgment prediction. Although the existing methods have achieved good prediction effect, the accuracy is still difficult to be greatly improved, mainly because the legal judgment prediction task still faces the following challenges:

1. There are topological dependencies among legal decision sub-data sets. An LJP usually consists of detailed and complex clauses, like the relevant legal provisions involved, the crime committed by the offender, and the level of punishment (fine, prison term, etc.). Therefore, the prediction of each subtask in a legal judgment should be a whole prediction, and there is interdependence among each task [13]. Zhong et al. [13] pointed out that for human judges, there is a strict order between the sub-data sets of legal decisions.
2. Sentence prediction based only on case description lacks prior knowledge. Compared with other sub-data sets, sentence prediction based on factual description is more challenging. In the real scene, when determining the sentence of a case, the judge will be influenced by many factors, including not only the age of the defendant described according to the facts of the case, the number of cases, but also the crime involved and other factors such as prior knowledge. Therefore, how to obtain the prior knowledge of sentence prediction under the supervision of the sub-data set information it depends on plays an important role in improving the final prediction performance. However, the existing sentence prediction task only makes prediction based on the fact description part of the case [14–16] or only considers the intermediate features of the sub-data sets it depends on in the training process as the prior knowledge of sentence prediction but lacks the process supervision of these prior knowledge [7, 9, 17].

To solve the above problems, this paper proposes a legal judgment prediction model (PS-LJP) based on process supervision. By considering the sequential topological dependence among various tasks, the prediction of relevant articles, crimes, and sentences in legal judgments is regarded as a sequential LJP problem. The process supervision information of each sub-data set is added in the training process so as to ensure the accuracy of the obtained information of the first task and then realize the effective prediction of the subsequent sub-data set. The model in this paper is based on the end-to-end recurrent neural network LJP framework. The supervision information of sub-data set labels is added to the LJP framework, and task-related features are expressed through the self-attention mechanism. The features of the prior task are taken as prior information and integrated with the features of subsequent tasks, and the result is used as the input of the subsequent prediction task to realize the decision prediction of sequential LJP.

## 2. Related Works

### 2.1. Prediction of Legal Decisions

Research on the prediction of legal judgments began many decades ago. Early studies were mostly limited by the limitations of public cases, and statistical-based methods achieved statistics for a small number of judgments rather than truly predicted [13, 18].

With the development of ML methods and NLP techniques, the legal judgment prediction task is regarded as a text classification task. Therefore, most legal judgment prediction tasks are specific to specific tasks, exploring how to extract more effective text features, which in turn achieve better crime prediction based on machine learning methods [9, 10, 17, 19, 20]. However, these traditional methods rely on hand-crafted shallow text features, with significant labor costs and poor domain adaptation, making it difficult to migrate to other scenarios.

Recently, DNN has been widely employed to [21] in the NLP field. Inspired by this, researchers try to integrate the deep neural network framework of legal knowledge for legal judgment prediction [7, 8, 13, 18, 22, 23]. For example, Luo et al. [12] adopted an NN method with attention mechanism to achieve the joint task of crime forecasting and related document extraction. Hu et al. [1–5] achieved the prediction of small sample and confusing crimes by defining 10 discriminative legal attributes. Ye et al. [6] use a sequence-to-sequence model to generate legal documents and realize crime prediction in civil cases. Zhong et al. [13] proposed the TOPJUDGE model, the first defining legal decision prediction as an LJP problem and proposed a topological LJP learning framework. However, without adding process supervision information, it is difficult to guarantee the accuracy of dependent features. Yang et al. [18] proposed an LJP learning framework that can encode multiple perspectives and multiple feedback on the dependencies and verification relationship between judgment sub-data sets, but this method is difficult to achieve end-to-end prediction and requires external auxiliary information.

### 2.2. Research Status of Text Classification

Traditional text classification methods are composed of feature engineering and classifier, in which feature engineering is used to extract feature information from text, and the classifier can obtain the probability distribution of each text category based on feature information. In the early text classification, bag of words, N-grams, and TF-IDF are usually used to extract features from the text, and then, support vector machine, naive Bayes, linear model, and K-nearest neighbor algorithms are combined to complete the text classification task. Word2vec tool is subsequently used to train the word vector. Each word in the text is represented as the word vector and used as the feature vector of the text. Different machine learning algorithms are used to achieve classification prediction. The text representation obtained by traditional text classification methods is usually high-latitude sparse vector, which cannot understand the deep semantic information in the text. Deep learning text classification method uses end-to-end training neural network model and can automatically extract semantic feature information from text. Experimental results show that text classification based on deep learning is generally better than the machine learning method. Joulin [24] proposed a fast and efficient text classification model (FastText), which uses the word bag (Bow) method to represent the whole sentence and constructs the relationship between text features and text categories by linear model. FastText is not only able to achieve the accuracy of other deep learning models but also significantly faster in training tests. Yoon et al. [25] proposed text classification model (TextCNN) based on convolutional network, which includes embedding layer, convolution layer, pooling layer, and full connection layer. Word vector has two modes: static and nonstatic. By using different sizes of filter layer and pooling layer, convolution text feature extracting method will reduce the dimension of the feature vector to make it more representative. The connection layer will effectively extract the text by giving the influence of different parameters on features according to the weight of classification features. Xiang et al. [26] constructed a character-based convolutional neural network model, which takes characters as the basic unit of sentence formation and does not require word segmentation in the text classification task based on the Chinese corpus, so as to avoid the situation of poor training model due to inaccurate word segmentation. Pengfei et al. [27] coded and represented texts with recurrent neural networks, trained multiple tasks simultaneously with an LJP learning framework, and modeled different text tasks using three different information-sharing mechanisms. Zichao et al.'s [28] multilevel attention model (HAN, hierarchical attention networks) adopts the bidirectional LSTM network in the words and sentences on the two levels to form different attention mechanism at the same time and has the ability to assign large weights to important words and sentences when constructing document representations. Siwei et al. [29] proposed a recursive convolutional neural network text classification model, using recursive structure to capture context information, and the maximum pooling layer in the convolutional neural network to determine which words play a key role in text classification so as to capture key elements in the text. Conneau et al. [30] paid attention to the influence of layers of the convolutional neural network on the classification effect, and the experimental results showed that increasing the number of convolutional layers was conducive to the extraction of more comprehensive text features.

### 2.3. Review of Similar Case-Matching Research

Similar case matching mainly compares the text similarity of two legal documents and selects the most similar one from the two candidate documents, which is a text similarity task in essence. However, due to the general description framework of legal documents and the professional words in the documents, higher requirements are put forward for similar case matching method. At present, most of the research on similar case matching is based on text similarity task, and the method is optimized according to the specific situation of the task. We then introduce the study of text similarity.

### 2.4. Review of Text Similarity Research

Text similarity is an important task in the field of natural language processing and has very important practical significance for other tasks, such as information retrieval, reading comprehension, and abstract generation. Early researchers proposed string-based methods by analyzing literal surface information in text. Representative methods include longest common substring, edit distance, and Jaccard. These methods simply consider the composition of characters or words and can generally be used for simple text similarity calculation tasks. Salton et al. [31] proposed a vector space model (VSM), and employed it to choose an optimum indexing vocabulary for a collection of documents. The evaluation results indicate the usefulness of the model. However, the document information of different words was counted and expressed in vector form by term frequency and inverse document frequency (TF-IDF); the disadvantage of this method is that the constructed text vector is usually high dimensional and sparse. The calculation efficiency is low. Landauer et al. [32] proposed the latent semantic analysis method (LSA), whose basic idea is to reduce the dimension of the high-dimensional sparse matrix represented by text by using singular value decomposition technology, so that the data finally obtained do not have high-dimensional sparsity and can better represent text information. Hofmann [33] improved the PLSA model based on LSA, and the model used maximum expectation algorithm to calculate text topic in LSA. Blei et al. [34] proposed an LDA topic model, whose basic idea is to use three different levels of the Bayesian model to model text topic, get text topic distribution through layer upon layer traversal, and calculate text similarity value by using this distribution. In recent years, deep learning techniques have been widely used in text similarity tasks. Mikolov et al. [35] proposed the Word2Vec word vector model tool. Word2Vec contains two different modes, CBOW or CSkip, to train the language model through shallow neural networks. Each word is represented as word embedding with general semantic information. On the basis of the word vector, each word in the text is represented as a fixed dimension vector, and the similarity of the text is calculated by calculating the similarity between the word vectors. Mikolov subsequently proposed the Doc2vec method [36], which is similar to the word vector representation method trained by Word2vec. Compared with word vector representation trained by Word2vec for a single word, Doc2vec can train word vector representation for the whole document. Doc2vec can avoid semantic deviation of the whole document caused by some inaccurate word vectors, so it has more advantages in the semantic representation of the whole document. Mueller et al. [37] proposed Siamse LSTM based on twin structure, which consists of two subrecurrent neural networks. Each recurrent neural network uses LSTM to encode and represent each text, and each text is represented as a vector of the same dimension. Finally, cosine similarity is used to calculate the similarity of two texts. Yin et al. [38] proposed a convolutional neural network (ABCNN) based on twin structure, which is used for sentence pair matching task. The model contains two subconvolutional neural networks, and an attention mechanism is added to the input layer and the convolutional layer of the convolutional neural network to better construct the semantic representation of text. Recently, Google researcher Devlin [39] proposed a pretraining model (Bert) based on bidirectional transformer encoder, which has the function of calculating the similarity of two texts. The training process includes pretraining and fine-tuning. Firstly, pretraining is carried out on large-scale unsupervised data so that the pretraining model has general semantic information. Secondly, the model is fine-tuned according to the specific task so that the model has the semantics of the specific task. The model has achieved breakthrough results in many natural language processing tasks.

This paper proposes a sequential LJP legal decision prediction model based on process supervision for end-to-end legal decision prediction. Different from the traditional LJP learning study on how to realize parameter sharing, the model in this paper not only models the sequential dependencies among various sub-data sets but also introduces a process supervision mechanism so as to realize the prediction of legal decisions by integrating prior information.

## 3. Data Processing

### 3.1. Feature Extraction Processing

Convolution neural network is one of the representative methods of deep learning technology, the convolutional neural network first began in the 1980s, and with the rise of artificial intelligence and machine computing power to ascend and the convolution neural network to get fast development, the different structures of convolution neural network are applied in computer vision, image processing, and other fields. A simple convolution neural network usually contains the input layer, convolution meter calculate layer, and pooling layer. The convolution meter calculation is the core of the CNN, which is used to extract local features of image or text information.

Researchers mainly mine text semantic features by constructing feature engineering and emotion dictionary, but they need to spend a lot of manpower on feature selection and design. In deep learning, the one-dimensional convolutional neural network CNN can obtain the local main semantic information of the text. Therefore, we used CNN network to extract features from the data in this paper. The structure of the CNN model includes three hidden layers in this paper as shown in Figure 1.

### 3.2. Dimension Reduction Processing

In the process of processing high-dimensional data in the model, important independent variables can be obtained by using variable selection, which can reduce the complexity of the model and ensure that the screened independent variables have a strong interpretation of the dependent variables. This method makes the model have the excellent performance of low-dimensional ideal model, so it has become a common method of scholars in various fields. The starting point of the variable selection method is summarized. First, the independent variable level is studied to test whether each independent variable can enter the model by establishing appropriate rules. These studies have formed traditional model selection algorithms based on AIC criterion, BIC criterion, RIC criterion, and so on. However, in the case of high dimensions, this kind of thinking is likely to fall into the dilemma of difficult calculation, that is, the frequently mentioned “dimension disaster” problem. PCA algorithm was proposed and widely used in various fields [40]. In our model, we will use the PCA algorithm to reduce the dimension of feature data.

## 4. A Computational Intelligence Model for Legal Prediction and Decision Support

In this paper, a sequential legal decision prediction model (PS-LJP) based on process supervision is proposed. The framework of the cyclic neural network which introduces process supervision is introduced.

### 4.1. Sequential Legal Decision Prediction Model (PS-LJP) Based on Process Supervision

This article proposes a sequence decision prediction framework based on process supervision, which consists of three layers: shared fact description coding layer, process supervision layer based on self-attention mechanism, and output prediction layer.

#### 4.1.1. Shared Fact Description Coding Layer

In the prediction framework adopted in this paper, the fact description coding layer is the shared layer of the prediction. For the description of facts, this paper adopts BiLSTM to encode the description of facts. To input, the LSTM unit calculates through the input gate, forgettable gate, update gate, and output gate and carries out characteristic coding on the input.

At each time step *t* ∈ [1, *n*], the LSTM unit takes *x*_*t*_ as the input, recalculates the storage unit *c*_*t*_, and outputs the new hidden state *h*_*t*_ as shown in the following equations:

(1) $$\begin{array}{c} f_{t}=\sigma \left(W_{f}\left[x_{t};h_{t-1}\right]+b_{f}\right). \end{array}$$

(2) $$\begin{array}{c} i_{t}=\sigma \left(W_{i}\left[x_{t};h_{t-1}\right]+b_{i}\right). \end{array}$$

(3) $$\begin{array}{c} o_{t}=\sigma \left(W_{o}\left[x_{t};h_{t-1}\right]+b_{o}\right). \end{array}$$

(4) $$\begin{array}{c} \hat{c_{t}}=\tanh\left(W_{c}\left[x_{t};h_{t-1}\right]+b_{c}\right). \end{array}$$

(5) $$\begin{array}{c} c_{t}=f_{t}\cdot c_{t-1}+i_{t}\cdot \hat{c_{t}}. \end{array}$$

(6) $$\begin{array}{c} h_{t}=o_{t}\cdot \text{tanh}\left(c_{t-1}\right). \end{array}$$

In the BiLSTM coding process, the forward LSTM network can obtain the left-to-right feature representation of the fact description, and the backward LSTM network can encode and fuse the semantics of subsequent features. Therefore, two hidden layer feature representation sequences $\left\{{\overset{⟶}{h}}_{1},{\overset{⟶}{h}}_{2},\cdots {\overset{⟶}{h}}_{n}\right\}$ and $\left\{{\overset{\leftarrow }{h}}_{1},{\overset{\leftarrow }{h}}_{2},\cdots {\overset{\leftarrow }{h}}_{n}\right\}$ and the two implicit states of each word are spliced together to obtain the implicit state representation $h_{j}={\overset{⟶}{h}}_{j};{\overset{\leftarrow }{h}}_{j}$ and finally obtain the following equation:

(7) $$\begin{array}{c} h=BiLSTM\left(x,\phi \right). \end{array}$$

In other words, the input vector *x* obtains high-level semantic output *h* through the coding of the BiLSTM network. Here, the dimension of the forward and backward implicit state is set as *d*/2, and the dimension of implicit state after splicing is set as *d*, and *ϕ* is the parameter involved in the above coding process.

#### 4.1.2. Process Supervision Layer Based on Self-Attention Mechanism

The process supervision layer based on the self-attention mechanism mainly introduces process supervision to obtain effective prior task-related dependency information, thus providing an important feature guarantee for subsequent sequential LJP dependency information fusion layer extraction. In the monitoring layer of the LJP process, the BiLSTM network based on the self-attention mechanism is adopted to obtain the fact description features of each sub-data set by using sub-data set label information to supervise.

Input the output *h* of the shared fact description coding layer into the BiLSTM network of |*T*| sub-data sets, respectively, and obtain the high-level semantic representation of each task:

(8) $$\begin{array}{c} h^{i}=BiLSTM\left(x,\phi_{i}\right),i=1,2,\cdots ,\left|T\right|, \end{array}$$

where *ϕ*_*i*_ is the parameter of BiLSTM corresponding to the *i* − *th* sub-data set. To better capture the relevant characteristics of each task, we introduce the attention mechanism by entering *h*^*i*^ into a full connection layer and mapping it between [0,1] using the softmax function.

(9) $$\begin{array}{c} a^{i}=softmax\left(W_{i}^{p}h^{i}+b_{ai}\right). \end{array}$$

Then, the feature representation for each sub-data set classification is obtained by weighted sum based on self-attention weight.

(10) $$\begin{array}{c} {\hat{h}}^{i}=h^{i}\cdot a^{i}. \end{array}$$

In order to ensure that each sub-data set can obtain its related feature representation from the fact description feature in modeling, category labels of each sub-data set are added for process supervision during this part of training, namely,

(11) $$\begin{array}{c} {\hat{y}}_{pi}=\text{soft }\max\left(W_{i}^{p}{\hat{h}}^{i}+b_{i}^{p}\right). \end{array}$$

Based on the obtained prediction result ${\hat{y}}_{pi}$, the minimum cross-entropy between ${\hat{y}}_{pi}$ and *y*_*pi*_ is adopted.

(12) $$\begin{array}{c} L_{pi}\left({\hat{y}}_{pi},y_{pi}\right)=-\overset{\left|Y_{i}\right|}{\underset{k=1}{\sum }}y_{pi,k}\log\left({\hat{y}}_{pi,k}\right). \end{array}$$

Process supervision is introduced to ensure that it can obtain effective sub-data set-oriented feature representation, which can guarantee the accuracy of sequential LJP prediction based on the dependency feature.

#### 4.1.3. Output Prediction Layer

Based on the feature representation *h*_*dj*_ of fusing dependent task information, it is linearly transformed and the final prediction of the task containing dependent information is realized by the softmax function so as to minimize the cross-entropy of the task containing dependent information.

(13) $$\begin{array}{c} {\hat{y}}_{dj}=\text{soft }\max\left(W_{j}^{d}{\hat{h}}^{j}+b_{j}^{d}\right),\\ L_{dj}\left({\hat{y}}_{dj},y_{dj}\right)=-\sum_{k=1}^{\left|Y_{i}\right|}y_{dj\;,k}\log\left({\hat{y}}_{dj\;,k}\right). \end{array}$$

#### 4.1.4. Training

For all prediction tasks, we weighted the sum of the process-supervised cross-entropy loss of each sub-data set and the final cross-entropy of the task containing dependent information so as to obtain the final loss function.

(14) $$\begin{array}{c} L=\sum_{i=1}^{\left|T\right|}\alpha_{i\cdot pi}\left({\hat{y}}_{pi},y_{pi}\right)+\sum_{j=1}^{\left|T\right|}\beta_{j\cdot dj}\left({\hat{y}}_{dj},y_{dj}\right), \end{array}$$

where *α*_*i*_ is the weight coefficient of each sub-data set in the process of process supervision and *β*_*j*_ is the weight coefficient of each sub-data set in the training process containing dependent information. In practice, we keep the weight of the loss function of process supervision and the weight of the sub-data set containing dependent information consistent. We only need to obtain the weight proportion of the two parts. Here, GA is used for parameter optimization.

## 5. Experiment

### 5.1. Data Set

The law prediction task uses the China Judicial AI Challenge data set CAIL2018, which is the first large-scale Chinese data set for predicting legal decisions. The data come from real criminal cases published by the Supreme People's Court. Each sample is judged by the factual description of the case and the corresponding outcome. In actual cases, many involve more than one defendant, which will greatly increase the difficulty of legal forecasting. Therefore, this paper only retains the sample of cases composed of a single defendant. According to statistics, the distribution of law categories in CAIL2018 is quite unbalanced. Some common crimes, such as theft and intentional injury, account for a large proportion. The data of the ten laws with the highest frequency account for 79.0% of the total data, while the data of the ten laws with the lowest frequency only account for 0.12% of the total data. The imbalance of data classes in CAIL2018 is a great challenge for the prediction of low frequency and obfuscation laws. The CAIL2018 data set consists of Small_CAIL2018 and Large_CAIL2018 data sets. Small_2018 contains 196,000 instrument samples, and Large_2018 contains 1.5 million instrument samples. The division of the two data sets in the experiment is shown in Table 1. In addition, we supplemented the CAIL2019 database to further verify the validity of our proposed model.

We use accuracy (Acc.), macro average precision (MP), macro average recall rate (MR), and macro average F1 value (F1) as evaluation indexes, where the macro average indicator refers to the average of all categories of indicators.

### 5.2. Experimental Results and Analysis

This article evaluates the prediction effect of four sub-data sets of legal judgment prediction: CAIL2018_Small, CAIL2018_Large, CAIL2019_Small, and CAIL2019_Large. To compare the experimental results, the following three models were used as the baseline models (each baseline system was trained under the LJP frame, and the best experimental results were compared):

1. *CNN*. In the text, the CNN model [15] containing multiple filter lengths is used to characterize and classify the fact description
2. *HSLTM*. Referring to the hierarchical neural network structure adopted by Yang et al. [41] in the emotion classification task, this paper adopts LSTM to encode sentence features and another LSTM to encode document features described by facts
3. *TOPJUDGE*. Zhong et al. [13] proposed a legal decision prediction model considering topological dependency among various sub-data sets, in which the representation of fact description features was obtained by LSTM coding

Tables 2–4 list the experimental results of the pretest for the four sub-data sets. The experimental results show that the PS-LJP model adopted in this paper outperforms the baseline system in four classification indexes of four data sets, which demonstrates the effectiveness of the model presented in this paper. Tables 2–5 list the experimental results.

It can be seen from Tables 2–5 that, (1) in the four data sets, all the models perform better in the Small data set than in the Large data set, which indicates that the size of the data set will directly affect the prediction accuracy of our method; (2) in the benchmark model and our proposed model, our model outperforms the benchmark model in the four data sets. This shows that our proposed model is better than some classical benchmark models for predicting legal decisions; (3) in general, compared with the single LJP, the PS-LJP model proposed by us has better performance in four different indicators on four data sets; (4) compared with the PS-LJP model without feature data preprocessing, the PS-LJP model based on principal component analysis proposed by us achieved better results in our four data sets.

More importantly, we found that the PCA-PS-LJP model we proposed achieved the best prediction results among all the models, which will prove that the method we proposed is very effective.

## 6. Conclusion

As an important subtask of intelligent justice, the study of law prediction is of great value. It can not only help legal personnel to deal with cases and improve work efficiency but also help ordinary people to understand cases and make them have certain psychological expectations for the outcome of cases. Based on the research of law prediction in intelligent justice, this paper analyzes the problems from the judicial perspective and converts them into text processing tasks. It adopts the deep learning technology to construct different neural network models and conducts training and testing on the basis of real legal data sets. In the law prediction task in this article, convolutional neural network (CNN) algorithm was used to extract text features, and the principal component analysis (PCA) algorithm was used to reduce the dimension of data features. Next, the prediction model based on process supervision is proposed for the first time. When modeling the dependency relationship between sequential sub-data sets, process supervision is introduced to ensure the accuracy of the obtained dependency information, genetic algorithm (GA) is introduced to optimize the parameters so as to improve the final prediction performance. Compared to our benchmark method, our algorithm achieved the best results on four different legal open data sets (CAIL2018_Small, CAIL2018_Large, CAIL2019_Small, and CAIL2019_Large).

## Figures and Tables

**Figure 1:** The structure of CNN model.

**Table 1:** Statistic information of CAIL2018 data sets.

Data sets	Small	Large
Training	150000	1450000
Test	30000	30000
Valid	16000	20000

**Table 2:** Prediction results of CAIL2019_Large.

Methods	Data set	CAIL2019_Large			
		Acc.	MP	MR	F1
Baselines	CNN	0.8219	0.8543	0.8836	0.8176
	HLSTM	0.8443	0.878	0.8082	0.8418
	TOPJUDGE	0.8444	0.8892	0.8015	0.8433

Ours	LJP	0.8453	0.884	0.8064	0.8436
	PS-LJP	0.8568	0.878	0.8368	0.57
	PCA-PS-LJP	0.8791	0.8786	0.8726	0.8682

**Table 3:** Results of CAIL2019_Small.

Methods	Data set	CAIL2019_Small			
		Acc.	MP	MR	F1
Baselines	CNN	0.8552	0.8765	0.8967	0.827
	HLSTM	0.8776	0.9002	0.8213	0.8512
	TOPJUDGE	0.8777	0.9114	0.8146	0.8627

Ours	LJP	0.8786	0.9162	0.8195	0.853
	PS-LJP	0.8901	0.9002	0.8499	0.8794
	PCA-PS-LJP	0.9124	0.9008	0.8857	0.8776

**Table 4:** Prediction results of CAIL2018_Large.

Methods	Data set	CAIL2018_Large			
		Acc.	MP	MR	F1
Baselines	CNN	0.8374	0.8742	0.8955	0.8361
	HLSTM	0.8698	0.8979	0.8201	0.8603
	TOPJUDGE	0.8599	0.9091	0.8134	0.8618

Ours	LJP	0.8608	0.9139	0.8283	0.8621
	PS-LJP	0.8723	0.8979	0.8487	0.8785
	PCA-PS-LJP	0.8946	0.8985	0.8845	0.8867

**Table 5:** Prediction results of CAIL2018_Small.

Methods	Data set	CAIL2018_Small			
		Acc.	MP	MR	F1
Baselines	CNN	0.8717	0.8876	0.9288	0.8488
	HLSTM	0.8951	0.9113	0.8534	0.873
	TOPJUDGE	0.8942	0.9125	0.8467	0.8745

Ours	LJP	0.8951	0.9173	0.8616	0.8748
	PS-LJP	0.9066	0.9113	0.882	0.9012
	PCA-PS-LJP	0.9289	0.9119	0.9178	0.8994

## Data Availability

Original data can be accessed through the following website: https://github.com/thunlp/CAIL.
